RETRACTED

# Small interfering RNA targeted to stem-loop II of the 5' untranslated region effectively inhibits expression of six HCV genotypes

**DOI:** 10.1186/1743-422X-3-100

**Published:** 2006-11-27

**Authors:** Ramesh Prabhu, Robert F Garry, Srikanta Dash

**Affiliations:** 1 Department of Pathology and Laboratory Medicine, Tulane University Health Sciences Center, 1430 Tulane Avenue, New Orleans, LA-70112, USA; 2 Department of Microbiology and Immunology, Tulane University Health Sciences Center, 1430 Tulane Avenue, New Orleans, LA-70112, USA

## Abstract

**Background:**

The antiviral action of interferon alpha targets the 5' untranslated region (UTR) used by hepatitis C virus (HCV) to translate protein by an internal ribosome entry site (IRES) mechanism. Although this sequence is highly conserved among different clinical strains, approximately half of chronically infected hepatitis C patients do not respond to interferon therapy. Therefore, development of small interfering RNA (siRNA) targeted to the 5'UTR to inhibit IRES mediated translation may represent an alternative approach that could circumvent the problem of interferon resistance.

**Results:**

Four different plasmid constructs were prepared for intracellular delivery of siRNAs targeting the stem loop II-III of HCV 5' UTR. The effect of siRNA production on IRES mediated translation was investigated using chimeric clones between the gene for green fluorescence protein (GFP) and IRES sequences of six different HCV genotypes. The siRNA targeted to stem loop II effectively mediated degradation of HCV IRES mRNA and inhibited GFP expression in the case of six different HCV genotypes, where as siRNAs targeted to stem loop III did not. Furthermore, intracytoplasmic expression of siRNA into transfected Huh-7 cells efficiently degraded HCV genomic RNA and inhibited core protein expression from infectious full-length infectious clones HCV 1a and HCV 1b strains.

**Conclusion:**

These *in vitro *studies suggest that siRNA targeted to stem-loop II is highly effective inhibiting IRES mediated translation of the major genotypes of HCV. Stem-loop II siRNA may be a good target for developing an intracellular immunization strategy based antiviral therapy to inhibit hepatitis C virus strains that are not inhibited by interferon.

## Background

Hepatitis C virus (HCV) is a major blood-borne human pathogen [1]. It is estimated that more than 170 million people worldwide have been infected with hepatitis C [2]. The majority of infected individuals develop life long chronic infections since only a fraction of people infected with HCV develop immunity and clear the virus infection [3]. Chronic hepatitis C virus infection can results in long-standing inflammation in the liver, which can lead to liver cirrhosis and hepatocellular carcinoma [4,5]. The only therapy currently available for HCV infection is the combination of interferon alpha and ribavirin. This therapy can effectively clear the virus infection in only a fraction of infected individuals. In the majority of patient infected the virus either does not respond to therapy or relapses when the therapy is discontinued [6-8]. Studies from our laboratories and others suggest that interferon inhibits hepatitis C virus replication by blocking it at the level of IRES mediated translation [9]. Therefore, the development of innovative approach to inhibit IRES may offer an alternative therapy for chronic hepatitis C patients that are non-responders to interferon.

RETRACTED

HCV is a positive-stranded RNA virus that belonging to the family *Flaviviridae *[10]. The HCV genome is approximately 9600 nucleotides in length and contains highly conserved 5' and 3' untranslated regions (UTR). These regions flanks a single large open reading frame (ORF) that encodes a large poly-protein processed into three different structural and seven nonstructural proteins. [11]. The highly conserved 5' UTR and 3' UTR sequences are required for both protein translation and virus replication [12,13]. The replication cycle of HCV occurs in the cytoplasm of infected cells making an excellent target for siRNA based antiviral development.

Since many individual cannot eradicate the virus infection with interferon based combination therapy, there is great interest to use this siRNA based antiviral strategy to treat a chronic HCV infection. A number of laboratories including our own have shown that siRNA targeted to the protein coding areas of HCV can inhibit virus replication and expression [14-21]. However, these viral coding sequences may not be the best target since they show significant variation among different HCV genotypes as well as virus sub-types. The nucleotide sequences of genomes from HCV isolated from different parts of the world vary considerably and are quite heterogeneous. Six major genotypes and more than 50 sub-types of the HCV virus have been described around the world. There are 30–50% variation in the nucleotide sequences among viral genotypes and 15–30% among different sub-types [22,23]. Isolates of HCV from a single patient can show 1–5% differences in their nucleotide sequences. In the United States, 75% of chronic hepatitis C cases belong to genotype 1a and 1b, 13–15% genotype 2a and 2b and 6–7% genotype 3a [24]. Genotype 1a and 1b is common in Western Europe. Genotype 3 is most frequent in the Indian subcontinent. Genotype 4 is the most common genotype in Africa and the Middle East. Genotype 5 is found in South Africa. Genotype 6 is found in Hong Kong and Southeast Asia [25]. Therefore, selection of siRNA targeted to a highly conserved region may be appropriate for developing a rational antiviral strategy against different HCV strains.

RETRACTED

In this study, we designed the most effective siRNAs targets in the highly conserved 5' UTR of the HCV genome. Their antiviral effect on IRES mediated translation was evaluated using sub-genomic clones and full-length infectious clones. We showed here that siRNA targeted to a unique location in the stem loop-II of 5' UTR inhibits IRES function of different genotypes and silence expression of multiple HCV genotypes.

## Results

### Intracellular delivery of siRNA inhibits GFP expression from HCV-IRES

Four different siRNAs (siRNA-74, siRNA-174, siRNA-207 and siRNA-245) targeting the 5' untranslated region (5'UTR) of hepatitis C virus genome were selected. The location and nucleotide sequence representing the RNAi target sites with respect to the predicted secondary structure of HCV IRES are shown in Fig. 1. pSuper-retro vector was used for intracellular production of siRNA in a liver derived cell line. Efficient transcription of siRNA from this vector occurs by host cell RNA polymerase using the H1-RNA gene promoter. As a negative control for our experiments, we used siRNA targeted to EBNA1 region of EBV. The effects of siRNA on the expression of green fluorescence protein from the IRES clones were examined by co-transfection experiments in Huh-7 cells. Initially, transfection experiments were performed to determine the optimum ratio of pSuper-retro siRNA and HCV IRES GFP plasmid for obtaining maximum inhibition of GFP from the IRES 1b clone. A ratio of 1:4 (one 100 nanogram of HCV-IRES-GFP and 400 nanogram of siRNA plasmid) produced the maximum inhibition. Using a similar experimental condition, the antiviral effect of four different siRNA targets on translation of individual HCV IRES GFP chimeric clone was examined. The specific inhibitory effect of siRNA on GFP expression was quantitated by flow cytometry analysis. The silencing of green fluorescence expression from different HCV IRES clones by four different siRNAs constructs is shown in Fig. 2. The siRNA-74 targeted to the stem loop II of HCV IRES was most efficient and completely silenced the expression of GFP in the case of all genotypes of HCV tested, siRNA-174 and siRNA-207 were moderately effective and siRNA-245 was the least effective. All three siRNA 74,174 and 207 effectively silenced expression of GFP from HCV 1a and HCV1b genotypes. These are the two most common genotypes of HCV in the United States that frequently develop resistance to interferon and ribavirin combination therapy. A control siRNA targeted to the Epstein Barr Virus nuclear antigen 1 (EBNA1) did not inhibit GFP expression in these experiments, indicating that the antiviral action of siRNA mediated gene silencing is highly specific. The numbers of GFP expressing Huh-7 cells after siRNA transfection was quantitatively measured by flow analysis (Fig. 3). It was determined that siRNA74 inhibited the IRES-GFP expression in approximately 80 to 90% of transfected Huh-7 cells in the case of all genotypes of HCV. Other siRNAs 174, 207 and 245 transfection inhibited GFP expression in only 40–60% of cells. The control siRNA specific to EBNA1 did not have any effect on GFP expression.

RETRACTED

**Figure 1:** Location of siRNA targets to the 5'UTR of HCV genome. Predicted secondary structure of the 5' UTR sequences (18–357). The sequence shown is that of the genotype 1a 5'UTR, HCV-H [40], and the structure based on previous studies [41-43]. Stem-loop structures are labeled for reference. The chimeric clones were made by fusing the GFP-encoding sequence, including a poly (A) tail, after the CCU sequence of the 5'UTR by overlapping PCR. The locations of siRNA targets in the stem-loop regions are shown by arrows.

**Figure 2:** Effect of small interfering RNAs on the expression of green fluorescent protein from IRES clones of six different HCV genotypes. Huh-7 cells were co-transfected with HCVIRES-GFP plasmid with siRNA plasmid (pSuper-retro) by using the FuGENE 6 transfection reagent. After 48 hours transfected cells were observed under a fluorescence microscope. The experiments were repeated for each genotype IRES clones using different siRNA constructs. SiRNA-74 was the most effective and inhibited the expression of green fluorescence in all genotypes of HCV compared to other siRNA. Control siRNA targeted to EBNA1 had no effect on GFP expression from HCV IRES clones.

**Figure 3:** Quantitative measurement of GFP positive Huh-7 cells by flow cytometry after siRNA transfection. Huh-7 cells were co-transfected with HCVIRES-GFP plasmid with siRNA plasmid (pSuper-retro) by using the FuGENE 6 transfection reagent. After 48 hours of transfection, cells were harvested and GFP positive cells were analysed by a flow cytometer (Becton Dickinson, BD Biosciences, Clontech). Percentage of GFP-positive Huh-7 cells was quantitatively determined after siRNA transfection using cell quest computer software. The results were expressed as percentage of control. siRNA-74 was found to be most effective in silencing GFP from all IRES clones.

### Intracellular delivery of siRNA74 inhibits expression of full-length clones of HCV 1a and 1b

The majority of chronic hepatitis C patients in the US are infected with HCV 1a or HCV1b genotypes, two genotypes of HCV that frequently develop resistance to interferon and ribavirin combination therapy. We tested whether this highly effective siRNA-74 target in the 5' UTR region could silence the gene expression using full-length infectious clones of HCV1a and HCV1b. One HCV1a infectious clone (pCV-H77C) and two HCV1b infectious clones of HCV (pMO9.6-T7 and pCVJ4L6S) were used as targets [26-28]. To examine the antiviral effect of siRNA-74, each full-length clone were co-transfected with increasing concentration of siRNA plasmid using a two-step transfection procedure described earlier (37–38). The inhibition of core protein expression of full-length clones of HCV 1a and HCV1b due to siRNA transfection was determined by immunoperoxidase staining (Fig. 4). Complete silencing of core protein expression was seen in Huh-7 cells transfected with HCV full-length clone 1a (pCV-H77C) and 1b (pMO9.6-T7 and pCVJ4L6S). This effect appears to be very specific since cells transfected with control siRNA targeted to EBNA1 silencing of core protein was not observed. Protein lysates were made and Western blot analysis was performed using the same monoclonal antibody specific for the HCV core protein. These results suggest that siRNA-74 effectively silenced gene expression from infectious full-length clones of HCV1a and HCV1b genotypes(Fig. 5). We then examined whether the silencing of core protein expression in the transfected cells caused intracellular degradation of HCV genomic RNA. Total RNA was isolated from the transfected cells and digested with DNaseI to eliminate plasmid DNA carryover from the transfection. The levels of positive strand HCV RNA were measured by ribonuclease protection assay (RPA). The results shown in suggest that siRNA74 degraded HCV positive- strand HCV RNA in a dose dependent manner in all clones (Fig. 6). Specificity of this silencing mechanisms occurring due to intracellular RNA degradation was examined by measuring HCV RNA levels in the cells co-transfected with control siRNA (EBNA1). These differences are not due to the variation of HCV RNA in the nucleic extracts since GAPDH mRNA levels are comparable in all samples. Taken together the results of our analysis suggest that siRNA-74 targeted to the 5'UTR region can inhibit IRES mediated translation of HCV and also are highly effective in silencing the gene expression of HCV 1a and HCV 1b strain.

RETRACTED

**Figure 4:** Immunocytochemical staining showing the silencing of core protein from full-length clones of HCV by siRNA-74. Huh-7 cells were co-transfected with (10 μg) pSuper-retro-siRNA74 and (10 μg) full-length clones of HCV. After 48 hours, transfected cells were harvested by the treatment with trypsin-EDTA. Cells were washed with PBS and immobilized onto a glass slide by cytospin method. Then slides were blocked and stained with core antibody against HCV using a mouse monoclonal antibody. Immunostaining for HCV core protein was performed using a standard protocol. The expression of core protein of full-length HCV 1a (pCVH77C), Ib (pCVJ4L6S), and 1b (pMO9.6--T7) is observed in the presence of siRNA74 and siRNAEBNA1 (unrelated siRNA).

**Figure 5:** Western blot analysis showing the silencing of core protein from full-length clones of HCV by siRNA transfection. Huh-7 cells were co-transfected with pSuper-retro-siRNA74 and full-length clones of HCV using the FuGENE 6 reagent. After 48 hours, transfected cells were isolated by the treatment with trypsin-EDTA. Cells were washed once with PBS and protein lysates were prepared and electrophoresed on 10% SDS-PAGE gels. The proteins were transferred to nitrocellulose membranes, blocked and immunoreacted with a primary antibody. The membrane was washed and incubated with peroxidase labeled secondary antibody and developed by ECL-chemiluminescence method. siRNA74 inhibited the expression of core protein in the case of all three full-length clones of HCV 1a and 1b. Beta actin levels were used as a control to make sure that equal amount of protein was present in the extracts.

**Figure 6:** Ribonuclease protection assay showing siRNA expression specifically degraded intracellular HCV positive strand RNA in the transfected Huh-7 cells. Huh-7 cells were co-transfected with different concentration of siRNA74 with different full-length clones of HCV. After 48 hours, transfected cells were isolated by the treatment with trypsin-EDTA. Total RNA was isolated and subjected to RPA for positive strand HCV using a minus strand RNA probe targeted to the 5'UTR region. The degradation of HCV positive strand by siRNA74 is concentration dependent. No HCV RNA degradation was observed in the cells transfected with unrelated siRNA.

## Discussion

Chronic HCV infection usually treated with a combination of pegylated interferon-alpha and ribavirin. However, the majority of chronic hepatitis C patients in the United States develop cellular resistance to interferon therapy. There is a need to develop new antiviral approaches to inhibit HCV replication. At present, there are several antiviral strategies that have been employed to inhibit HCV virus replication [29]. Among these, RNA interference appears to be one of the most powerful antiviral approaches to inhibit HCV gene expression in mammalian cells. RNA interference (RNAi) is a sequence specific RNA degradation process in the cytoplasm of eukaryotic cells induced by double-stranded RNA [30,31]. This process can be initiated via so called small interfering RNAs (siRNA) of approximately 19–23 base pairs. These are cleaved by double-stranded precursor RNAs by the RNase III-like enzyme dicer. These siRNAs associate with various proteins to form the RNA-inducing silencing complex (RISC), harboring nuclease and helicase activity. The antisense strand of the siRNA guides the RISC to the complementary target RNA and the nuclease component cleaves the target RNA in a sequence specific manner. This approach has been a widely used as a technique for gene knockouts for gene expression studies and as an antiviral against a number of viruses [32-34]. The RNAi approach is very specific and offers a great potential to be used as antiviral against hepatitis C virus infection. Reports from the previous studies including our own experience suggest that this siRNA-based approach is very effective by yielding up to 100-fold inhibition of virus replication [14-20]. We have used siRNA targets in the E2, NS3 and NS5B region and showed that these siRNA targets can silence HCV 1a infectious clone effectively. However, the same siRNA does not work effectively against other viral strains, because of sequence variation in the siRNA target. To develop siRNA targets that can be used for both HCV 1a and HCV1b virus and other genotypes we selected the highly conserved region of HCV. The 5' untranslated region (UTR) of HCV consisting of 341 nucleotides, is highly conserved among different viral genotypes and in clinical strains of HCV [35]. We selected four siRNA targets in the second and third stem-loop regions of secondary structure of 5'UTR. To direct the synthesis of fully processed siRNA-like transcripts in transfected Huh-7 cells a mammalian expression plasmid vector (pSuper-retro) was used. The use of the vector-based delivery is more efficient because it allows continuous transcription of siRNA in the transfected cell. We showed that intracellular expression of siRNA silences GFP expression from IRES clones. Some of the siRNA targets appear to be more efficient than others. For example, siRNA-74 is found to be most effective against six different viral IRES sequences as compared to the other three. The siRNA-174, siRNA-207 is moderately effective against HCV 1a and HCV 1b IRES. The siRNA-254 was the least effective against HCV1a and HCV1b IRES, but it was highly effective against 2b, 3a, 4a IRES. The results could be due to the fact that there are some nucleotide variations in the IRES sequences among different virus genotypes. There are also published reports suggesting that many cellular proteins binds to the 5' UTR sequence of HCV for translation of polyprotein. It is possible that the some siRNAs could not have efficiently hybridize to some sequences in the transfected cells than the others because of complex secondary structure of the 5'UTR.

RETRACTED

We extended this study and examined whether the siRNA-74 could also effectively silence gene expression of HCV 1a and 1b strain. We used full-length chimpanzee infectious clones as viral targets. The full-length HCV genomic clone was expressed in Huh-7 cells by the use of adenovirus T7 RNA polymerase. We have shown that this inducible model allows high-level expression of HCV structural and non-structural proteins that can be measured by Western blot analysis (37,38). Replication of HCV full-length genome 1a and 1b was observed in the transfected hepatic cell lines by detecting viral negative strand RNA by strand specific ribonuclease protection assay. Using co-transfection studies, it was determined that complete silencing of HCV core protein expression was observed by siRNA-74 for HCV 1a and HCV 1b infectious clones. The inhibition of viral protein expression by siRNA-74 was confirmed by an immunocytochemical method as well as by Western blot analysis. No inhibition was seen in the cells co-transfected with unrelated siRNA, suggesting that the antiviral effect of siRNA-74 is specific. These results were confirmed by looking at the stability of full-length HCV genomic RNA in the transfected cells by RPA. Silencing of the viral protein expression was due to the specific degradation of HCV genomic mRNA. Our results clearly support the hypothesis that the siRNA-74 can cause gene silencing of HCV1a and HCV1b strains. In summary, these results clearly show that the siRNA mediated viral gene silencing is a very effective antiviral strategy that has a very strong potential for curing chronic hepatitis C virus infection. The siRNA-74 is an important therapeutic target for the treatment of infection of multiple genotypes of HCV.

## Conclusion

In the present study we identified a siRNA targeted to the stem loop II (siRNA-74) of 5'UTR of HCV that inhibited the expression of GFP in six different chimeric clones of HCV as well as inhibited the expression of the core protein and degraded the positive strand RNA in full-length clones of HCV 1a and 1b. Therefore, our results support that use of the siRNA74 as an important target for inhibiting IRES mediated translation of multiple genotypes of HCV.

## Methods

### Cell line and Transcription plasmid

Huh-7 cell line was maintained in Dulbecco's Modified Media (D-MEM) containing non-essential amino acids, sodium pyruvate and 10% fetal bovine serum (In vitrogen Life Technologies, Carlsbad, CA). Chimeric clones between IRES sequences of six different HCV genotypes and green fluorescence protein used here were constructed previously [36]. A chimpanzee infectious clones pCV-H77C (HCV1a) was obtained from Jens Bukh, National Institute of Health [26,27]. Full-length HCV transcription plasmid (pNIH1a-Rz) was prepared using chimpanzee infectious clone (pCV-H77C), which contains a T7 promoter, full-length cDNA of HCV genome, followed by a cDNA copy of autolytic ribozyme from antigenomic strand of hepatitis delta virus and T7 transcriptional terminator sequences. Detailed description of transcription plasmid and method has been described previously [37,38]. A chimpanzee infectious clone (pCVJ4L6) was obtained from Jens Bukh, National Institute of Health. Transcription plasmid (pTRE-NIH1b) was prepared by addition of hepatitis delta virus ribozyme sequences and T7 transcriptional terminator at the very end of 3'UTR using the methods described in our publications. A chimpanzee infectious clone pMO9.6-T7 (HCV1b) containing an autolytic ribozyme sequence from antigenomic strand of hepatitis delta virus and T7 transcriptional terminator sequences at the 3' end was used here as described previously [37,38].

RETRACTED

### Construction of pSuper-retro vector encoding siRNAs

Four different siRNAs were selected and targeted to the 5' UTR region of HCV genome (1b) using web-based Oligo-Engine software. As a control, siRNA targeted to Epstein barr virus (EBV) nuclear antigen was used [39]. A commercially available plasmid vector called pSuper-retro (Oligo- Engine) for intracellular delivery of siRNA was used. The siRNA constructs were prepared at two steps. In the first step, we synthesized a pair of (sense and anti-sense orientation) 64-nts oligos containing 19 nucleotides of HCV in sense and antisense orientations, separated by a 9-nt spacer sequence. Restriction enzymes *Xho1 *and *Bgl II *were introduced at the 5' end of sense and antisense 64 nucleotide oligos for cloning. In the second step, the sense and antisense primers were annealed by incubation at 90°C for 4 min then 72°C for 10 minutes. The annealed oligos were then slowly cooled to 10°C and ligated to the pSuper-retro vector using *Xho1 *and *Bgl II *restriction sites. The nucleotide sequences of the sense and antisense primer used to design the siRNA vectors are shown in Table 1. The recombinant clones containing the iRNA insert were selected by restriction enzyme digestion. Large-scale plasmid DNA isolation was performed using a maxi kit (Qiagen Inc). The presence of siRNA sequences was confirmed by DNA sequence analysis.

RETRACTED

**Table 1:** Sequences of small interfering RNAs used to target the 5' UTR of hepatitis C virus RNA

Name of the siRNA	Nucleotide sequence
siRNA 74 S	5'-AGCGTCTAGCCATGGCGTT-3'
siRNA74 AS	3'-TCGCAGATCGGTACCGCAA-5'
siRNA174 S	5'-TTGCCAGGATGACCGGGTC-3'
siRNA174 AS	3'-AACGGTCCTACTGGCCCAG-5'
siRNA207 S	5'-CCCGCTCAATGCCTGGAGA-3'
siRNA207 AS	3'GGGCGAGTTACGGACCTCT-5'
siRNA245 S	5'-GACTGCTAGCCGAGTAGCG-3'
siRNA245 AS	3'-CTGACCATCGGCTCATCGC-5'

### Effect of siRNA on expression of GFP from different IRES clones

Huh-7 cells were grown in a 12- well tissue culture dish the day before transfection. The next day the cells were infected with a replicative defective adenovirus that expressed T7 RNA polymerase. After two hours, cells were co-transfected with 100 ng of HCV-IRES-GFP plasmid and different concentrations siRNAs plasmid using FuGENE 6 reagent (Roche Molecular Biochemicals, Indianapolis, IN). Expression of green fluorescence was recorded at 24, 48 and 72 hours using a fluorescence microscope. The ratio of IRES plasmid to siRNA-74 plasmid required for maximum inhibition of GFP expression from the IRES clone was recorded. Using the identical condition effect of four different siRNAs on GFP expression from IRES clone was examined. The inhibitory effects of each siRNA plasmid on GFP expression from six different HCV IRES sequences were quantitatively by flow analysis. Transfected cells were harvested by treatment with trypsin-EDTA, and then resuspended in PBS (Invitrogen Life Technology, Carlsbad, CA) and subjected to flow-cytometric analysis (Becton Dickinson, BD Biosciences Clontech). The percentage of GFP-positive Huh-7 cells was quantitatively compared with control siRNA for different siRNA with different HCV genotypes.

### Effect of siRNA on expression of full-length HCV genome

To examine the effect of siRNA on expression of full-length HCV 1a and 1b strain was examined by co-transfection experiments. We have developed a T7- based model in which expression of full-length HCV RNA genome can be reliably studied in Huh-7 cells. Detailed methodology has been described previously [37,38]. Huh-7 cells were co-transfected with 10 micrograms of HCV full-length plasmid and different concentration siRNAs plasmid using FuGENE 6 reagent. The success of intracellular delivery of each siRNA targets against full-length HCV 1a and HCV1b strain was examined by measuring core protein and positive strand HCV RNA.

### Immunoperoxidase Staining

The extent of core protein inhibition due to siRNA74 on full-length clones of HCV1a and 1b was examined by immunostaining of transfected Huh-7 cells using a monoclonal antibody (Affinity Bioreagents, Denver. CO). Transfected Huh-7 cells were immobilized onto glass slides by cytospin method. Cells were washed with phosphate-buffered saline (PBS) pH 7.4 twice, air-dried and fixed with chilled acetone for five minutes. The cells were permeabilized by treatment with 0.05% saponin for 10 minutes at room temperature. Blocking was performed with 5% normal goat serum (Sigma Chemical Company, St. Louis, MO) diluted in minimum essential medium for 30 minutes at room temperature. Blocking for endogenous biotin-avidin was performed using blocking reagents from the kit (Avidin/Biotin Blocking Kit, Vector Laboratories Inc., Burlingame, CA) and blocking for endogenous peroxidase was done with 0.9% H_2_O_2 _for 30 minutes at room temperature. The cells were incubated with monoclonal anti-core antibody (1:100 dilution) overnight at 4°C. The next day they were washed three times and incubated with anti-mouse biotin conjugated antibody (1:1000) for one hour at room temperature. The slides were washed and incubated for 30 minutes with Elite avidin-biotin peroxidase complex (VECTOR Labs, CA). The slides were then reacted with diaminobenzidine for 10 minutes and then counterstained with hematoxylin for one minute. After dehydration, the slides were mounted with permount and observed under light microscopy.

RETRACTED

### Western Blot Analysis

Western blot analysis for core protein was performed on protein lysate from transfected cells using a standard protocol in our laboratory [37,38]. Briefly, transfected cells were treated with 500 μl of lysis buffer containing 150 mM sodium chloride, 50 mM Tris-HCl, 1% NP-40, 0.5% deoxycholate, 0.1% SDS and protease inhibitors (Protease Inhibitor Cocktail, Roche Biochemicals, Indianapolis, IN). Fifty micrograms of the total cell lysate was separated by 10% SDS-PAGE and transferred onto nitrocellulose membranes (Amersham, Arlington Heights, and IL). The membranes were blocked with PBS containing 5% non-fat dried milk and 0.1% Tween-20 for 1 hour at room temperature. Then, the membrane was incubated with monoclonal antibody against core (Affinity Bioreagents, Denver, CO) at 1:100 dilutions for one hour. The membrane was washed three times with 0.1% Tween-20 in PBS. Following this step, the membranes were incubated with peroxidase-labeled secondary antibody (ECL Western blotting analysis system, Amersham Pharmacia Biotech UK, Amersham PLC, Buckinghamshire, England) at a dilution of 1:1000 for one hour. After this step, membranes were washed three times with PBS and developed using ECL Chemiluminescence Detection Kit (Amersham Pharmacia Biotech UK, Amersham PLC, and Buckinghamshire, England). To verify that equal amounts of protein were loaded onto each lane of the SDS-PAGE, the membrane was incubated with monoclonal antibody to beta-actin.

RETRACTED

### Ribonuclease Protection Assay (RPA)

Levels of HCV genomic RNA (positive strand) in the siRNA-transfected cells were examined by RPA. Total RNA was isolated from the transfected cells by the GITC method. RNA extracts were treated with DNase I (Roche Molecular Biochemicals, Indianapolis, IN) 5U/mg of RNA for one hour at 37°C to remove any residual plasmid DNA templates. RPA was performed to detect the presence of HCV-positive in transfected Huh-7 cells (Ambion, Austin, TX). The RNA probe targets the highly conserved 5' UTR of HCV genome. The plasmid pCR II-296 was linearized with *Xba I *and used to prepare an anti-sense RNA probe using the SP6 RNA polymerase in the presence of ^32^P-UTP. For RPA assays, approximately 1 × 10^6 ^cpm of the labeled anti-sense probe was added to 25 μg of RNA sample and vacuum dried. Hybridization was performed in 10 μl of the hybridization buffer after denaturing for 3 minutes at 95°C and followed by overnight incubation at 45°C. RNase digestion was performed in 200 μl of RNase cocktail (1: 100) (Ambion Inc. Austin, Texas) in a buffer consisting of 10 mM Tris, pH 7.5, 5 mM EDTA and 0.3 M NaCl for 1 hour at 37°C. Reactions were stopped by the addition of 2.5 μl of 25% SDS and 10 μl of proteinase K (10 mg/ml) at 37°C for 15 minutes. Samples were extracted with phenol/chloroform and precipitated with ethanol. The pellet was air dried and resuspended in 15 μl of gel loading buffer. The samples were then boiled for 3 minutes and separated on an 8% acrylamide/8 M urea gel. The gel was dried and exposed to X-ray film (Kodak, X-OMAT-AR).

## List of abbreviations

HCV, hepatitis C virus; RNAi, RNA interference; siRNA, small interfering RNA, dsRNA, double stranded RNA; IRES, internal ribosome entry site; GFP, Green fluorescence protein.

## Competing interests

The author(s) declare that they have no competing interests.

## Authors' contributions

All authors have contributed equally to the work presented in this paper.
